# Medical Intelligent System and Orthopedic Clinical Nursing Based on Graph Partition Sampling Algorithm

**DOI:** 10.1155/2022/2764157

**Published:** 2022-06-14

**Authors:** Xiucheng Heng, Yufei Chen, Lihong Liu

**Affiliations:** ^1^China Medical University, The Fourth Affiliated Hospital of China Medical University, Shenyang, Liaoning 110032, China; ^2^Department of Orthopedics, Air Force Medical Center of PLA Department of Orthopedics, The Fourth Medical Sciences, Beijing 100142, China

## Abstract

This study summarizes the process of graph partition sampling algorithm. Through studying, observing, and comparing many different types of graph partition sampling algorithms, this study represents the learning process sampling into three steps: sampling process, aggregation process, and the calculation process of loss function. The medical intelligence system developed in this study must provide remote audio and video connections between patients, nurses, and doctors, and requires hardware, software, and network collaboration. The hardware includes a server that keeps the medical intelligence system running. The software includes the operating system and server application software that provide the basic functions of the system. The network platform provides network bandwidth and basic configuration to achieve effective connections between different parts. At the same time, the system also defines audio and video encoding and decoding standards. Orthopedic patients are often accompanied by varying degrees of activity limitation and low self-care ability, the particularity of these patients puts forward higher requirements for orthopedic clinical care management. Orthopedic clinical nursing path is a standardized nursing management method supported by evidence-based medicine. In order to meet the requirements of the system design, the goal of the system design is to use the latest computing and network communication technology to organically “connect” the nursing staff, the nursing staff, and the hospital, so that the nursing staff can enjoy the personalized guidance specially made by the doctor at any time.

## 1. Introduction

In recent years, graph partition sampling algorithms map and encode the structure of graphs into low-latitude vector spaces, which have gradually attracted attention. This type of method is mainly based on deep learning, matrix decomposition, or nonlinear dimensionality reduction. The method based on deep learning makes the vector representation of the graph more accurate by introducing the node attribute vector [1]. However, in this scenario, the dimension of the node becomes higher and the scale of the graph becomes larger, and access to node attributes will become a training bottleneck. This study aims to optimize the existing algorithm based on the method of graph partition sampling algorithm. Ensure that the advantages of deep learning operators and node attribute vectors are fully utilized without reducing training performance. In the context of the continuous development of China's medical intelligent system, the drawbacks of the traditional medical model have gradually emerged. At present, most hospitals use doctors and nurse to inspect the patient's physical condition, and cannot monitor the patient's physical condition at any time [2, 3]. Although a patient can press a button to call a medical staff in an emergency, waiting for the medical staff to arrive at the ward before judging the patient's condition may cause a delay in diagnosis. On the basis of traditional medical diagnosis, many medical staff has put forward a new point of view, that is, we are currently in need of a new medical intelligent system. Clinical nursing path is a standard process of diagnosis and treatment with scientific and chronological characteristics [4]. This type of nursing method takes the past successful nursing experience as a reference, through a comprehensive summary and analysis, formulates the best nursing plan that meets the needs of the patient, and applies it to nursing practice [5]. In orthopedic clinical nursing, clinical nursing pathway intervention methods require orthopedic clinical nurses to jointly develop orthopedic nursing pathway tables, and in the process of implementing nursing management with reference to the pathway tables, promptly identify and discover the parts of the pathway tables that need improvement, and combine the actual conditions of the patients. It is necessary to make appropriate adjustments to the content of the path table to ensure the quality of care for orthopedic patients. The study describes the specific system design and implementation results of the system back-end management functions, the basic data operation functions of medical management, the real-time data transmission of intraoperative monitoring, and the real-time video transmission of intraoperative monitoring. The authority management framework is built through the RBAC model to achieve authority management in the system. Because medical data, especially patient-related data, are all private information, if the medical data leaks, it will not only affect the image of the hospital, but also affect the patients themselves. Therefore, the system design ensures the security of the accessed data by implementing https encryption, using md5 to encrypt and store the password, designing a signature verification mechanism to verify whether the parameters have been tampered with, and preventing CSRF attacks.

## 2. Related Work

The literature introduces how the overall framework of the intelligent medical monitoring service system is designed and how to divide the boundaries between microservices. It introduces how the database model is designed and the physical table structure that is finally mapped into it. Finally, it also introduces the metadata-driven content used in the data model design process. The literature introduces the detailed design plan and implementation of the back-end management function of the intelligent medical monitoring service system, the design and implementation of the core function, real-time data, and real-time video transmission in the system. Since the whole system is modularized by microservices, this chapter introduces event-driven way to achieve the realization of communication between services [6, 7]. The literature describes system optimization testing and deployment. In order to discover all kinds of errors or exceptions that exist or potential in the system before the official release, unit testing is necessary. Introduced the unit test methods and various test cases of each module, optimized the function of slow query problems in the test, and introduced how to use the master-slave server to achieve data disaster recovery processing, and finally introduced the rapid deployment of the entire system. The literature introduces the telemedicine system, which combines advanced medical technology with modern computer and communications technology [8]. A telemedicine system is based on JAVA multimedia framework and real-time transmission protocol. It supports functions such as telemedicine advice, medical care, emergency medical assistance, and medical advice, and has functions such as multimedia interaction, collaboration, and resource sharing suitable for nursing care [9, 10]. It can enable the nursing staff to communicate with medical staff in a timely and effective manner and provide medical convenience. The literature introduces research on telemedicine systems, explains the JMF and RTP protocols used in system development, and explains how to combine these two technologies for system design [11–13]. Then, the requirements of the telemedicine system are analyzed, and the overall structure is designed to analyze the functions and relationships of each module. Carefully studied the design of audio/video and client management subsystems, and finally used test cases to test and verify certain functions of the system.

## 3. Graph Partition Sampling Algorithm and Medical Intelligent System Model Design

### 3.1. Basic Principles of Graph Division

Before graph representation learning officially rose and became popular, the node classification tasks on the graph were mainly based on data analysis methods, such as matrix decomposition, or machine learning methods to analyze graphs. The input of this type of algorithm is the original data of the graph, such as the adjacency matrix of the graph. The analysis and calculation of matrices is a discipline with a very long history. The methods include matrix dimensionality reduction and extraction of eigenvectors of the matrix. Early methods also focused on the analysis of the adjacency matrix.

This method uses the feature matrix of *L* as the feature expression, and implicitly considers that the segmentation of the graph is valuable for accurate classification.

(1) $$\begin{array}{c} \tilde{ℒ}=D^{-1/2}{\text{LD}}^{-1/2}=I-D^{-1/2}{\text{AD}}^{-1/2},\\ L=D-A. \end{array}$$

In algorithms that use random walks to capture the structure of the graph, such as DeepWalk, after selecting a root node of the walk, the node sequence generated by the walk is nothing more than a combination of two search strategies on the graph: graph width priority search and image depth-first search. The process of random walk to generate random sequence is similar to depth-first search and breadth-first search, as shown in Figure 1.

Given the source node *u*, and the length of the random walk *l*, use ci to represent the *i*th node in the path, *C*_0_ = *u*. The probability of random walk transition is shown in (2), where *π*_*vx*_ is the transition probability that is not normalized, and *Z* is the normalization constant. In order to adjust different walking strategies for different applications, node2vec uses a biased search method. node2vec defines two parameters *p* and *q* to control the preference of wandering.

(2) $$\begin{array}{c} P\left(c_{i}=x|c_{i-1}=v\right)=\left\{\begin{array}{cc} \frac{\pi_{vx}}{Z}, & \mathrm{if}\left(v,x\right)\in E,\\ 0, & \mathrm{other}. \end{array}\right. \end{array}$$

*d*_*tx*_ represents the shortest distance from node *t* to node *x*.

(3) $$\begin{array}{c} \alpha_{pq}\left(t,x\right)=\left\{\begin{array}{cc} \frac{1}{p}, & \mathrm{if}\;d_{tx}=0,\\ 1, & \mathrm{if}\;d_{tx}=1,\\ \frac{1}{q}, & \mathrm{if}\;d_{tx}=2. \end{array}\right. \end{array}$$

For each source node *u* ∈ *V*, NS(*u*)∈*V* represents the set of neighbor nodes generated by the sampling of node *u*. The loss function of node2vec is shown in the formula.

(4) $$\begin{array}{c} \underset{f}{\max}\sum_{u\in V}\log\;\mathrm{Pr}\left(N_{S}\left(u\right)|f\left(u\right)\right). \end{array}$$

This symmetry is manifested in the formula, that is, the calculations of the nodes appear in pairs.

(5) $$\begin{array}{c} \mathrm{Pr}\left(n_{i}|f\left(u\right)\right)=\frac{\text{exp}\left(f\left(n_{i}\right)\right)\cdot f\left(u\right)}{\sum_{v\in V}\exp\left(f\left(v\right)\cdot f\left(u\right)\right)}. \end{array}$$

Taking the Pr(*n*_*i*_|*f*(*u*)) obtained based on the above assumptions into formula (4), the final objective loss function can be obtained as

(6) $$\begin{array}{c} \underset{f}{\max}\sum_{u\in V}\left[-\log\;Z_{u}+\sum_{n_{i}\in N_{S}\left(u\right)}f\left(n_{i}\right)\cdot f\left(u\right)\right]. \end{array}$$

### 3.2. Function Model

In machine learning, the loss function directly determines the direction of parameter learning. In traditional machine learning, multiple features can be added to the model by designing the loss function. In graph representation learning, the characteristics of these loss functions are also applicable, and the loss function directly determines the learning goal. In the supervised or semisupervised learning algorithm, the design of the loss function is much more flexible due to the existence of the label of the target node. For unsupervised learning, there is no clear learning goal for a given training sample. Therefore, the main algorithm currently used is to compare the training node with positive and negative samples. The goal of the loss function for training the model is to make the nodes in the training samples closer to the nodes in the positive samples and farther away from the nodes in the negative samples. The following describes the loss function in detail with regard to supervised semisupervised and unsupervised learning algorithms.

(7) $$\begin{array}{c} p_{1}\left(v_{i},v_{j}\right)=\frac{1}{1+\text{exp}\left(-{\overset{⟶}{u}}_{i}^{T}\cdot {\overset{⟶}{u}}_{j}\right)}. \end{array}$$

Then in the training process of the model, the most direct way to capture the structural information of the first-order distance is to minimize the objective function expressed by the following formula:

(8) $$\begin{array}{c} O_{1}=d\left({\hat{p}}_{1}\left(\cdot ,\cdot \right),p_{1}\left(\cdot ,\cdot \right)\right). \end{array}$$

Using relative entropy to represent the distance between probability distributions, the objective function can be obtained as shown in the following:

(9) $$\begin{array}{c} O_{1}=\sum_{\left(i,j\right)\in E}\omega_{ij}\log\;p_{1}\left(v_{i},v_{j}\right). \end{array}$$

The desired effect of the second-order distance is that for nodes that are not directly connected (that is, the first-order distance between nodes is zero), if the two nodes share many identical neighbor nodes, then the two nodes are at low latitudes. The expression in space should still be similar. Therefore, in the representation of the second-order distance, it should be noted that the node plays two different roles: the source node and the context node. Therefore, when nodes play different roles, they need to use different representation vectors to calculate the second-order distance between nodes.

(10) $$\begin{array}{c} p_{2}\left(v_{j}|v_{i}\right)=\frac{\exp\left({{\overset{⟶}{u}}^{\prime }}_{j}^{T}\cdot {\overset{⟶}{u}}_{i}\right)}{\sum_{k=1}^{\left|V\right|}\exp\left({u^{\prime }}_{k}^{T}\cdot {\overset{⟶}{u}}_{i}\right)}. \end{array}$$

Then the objective function to capture the second-order distance structure information is as shown in the formula:

(11) $$\begin{array}{c} O_{2}=\sum_{i\in V}\lambda_{i}d\left({\hat{p}}_{2}\left(\cdot |v_{i}\right),p_{2}\left(\cdot |v_{i}\right)\right). \end{array}$$

As with the first-order distance, relative entropy is used here to represent the distance between two probability distributions. Then the objective function to evaluate the second-order distance is shown in the formula:

(12) $$\begin{array}{c} O_{2}=\sum_{\left(i,j\right)\in E}\omega_{ij}\log\;p_{2}\left(v_{j}|v_{i}\right). \end{array}$$

In unsupervised learning scenarios, GraphSage requires a loss function based on the graph structure. The graph-based loss function allows adjacent nodes (positive samples) to have more similar expressions, while using isolated nodes (negative samples) to have a higher degree of discrimination, as shown in the following:

(13) $$\begin{array}{c} ℒ\left(z_{u}\right)=-\text{log}\left(\sigma \left(z_{u}^{T}z_{v}\right)\right)-N\cdot E_{v_{n}P_{n}\left(v\right)}\text{log}\left(\sigma \left(-z_{u}^{T}z_{v_{n}}\right)\right). \end{array}$$

### 3.3. Sampling Algorithm Data Set

Graphical data comes from real-world phenomena, such as social networks and the Internet. A typical feature is that the order of the nodes in the graph satisfies a power-law distribution, which is represented by connecting a small number of nodes to most nodes in the graph. For example, celebrities have more than 60 million fans, but most ordinary people have only hundreds of fans. The characteristics of this power-law distribution can easily cause a certain part of the data to overheat and cause the server to go down. For example, Sina Weibo often shows news that a celebrity announces their marriage, and then the entire server goes down.

This study takes PPI (Protein Interaction Network) and Reddit Forum Post Comment Network as examples to illustrate the universality of the power-law distribution of graphs from the perspective of real data sets. As shown in Figure 2, use the visualization tool to calculate the node degrees in the two data sets, and draw the relationship curve between the number of nodes and the node degrees. For these two types of actual records, they originate from two different fields, and there are long tail characteristics. A very small part of the nodes are connected to most of the nodes, and most of the nodes are associated with a small number of nodes, which also determines the sparsity characteristics of the graph structure. From the curves of these two real data sets, it can be seen that the characteristics of power-law distribution are reflected in many application scenarios and are universal.

This study optimizes the sampling algorithm based on the characteristics of vector learning and the power-law distribution of graphs. In fact, not all neighbor nodes are needed for neighbor sampling. Regardless of whether it is random walk sampling or sampling according to a certain probability distribution, for graph structures with power-law distribution characteristics, the neighbor list of nodes with high numbers will be truncated, while nodes with low degrees will be filled with existing neighbors. The schematic diagram is shown as the black rectangle in Figure 3. It can be seen from the figure that, for the nodes on the left, only a part of the nodes are taken as neighbor nodes that gather structural information. For the node on the right, because there are not so many neighbor nodes, the existing neighbor nodes are reused to complement.

Therefore, in this study, an algorithm for partitioning according to the degree is proposed, so that the sample-based unsupervised training corresponds to the attributes of the power law of the graph. According to the nature of the power-law distribution, the nodes can be sorted from high to low. Collect large nodes in a block, and make full use of the feature matrix of nodes in a block.  Figure 4 shows the result of dividing a typical graph that satisfies the power-law distribution.

In the actual data set, you can see that most of the edges are gathered around the node, which is the basis for optimizing the algorithm in this document. The key to making full use of the partition is to optimize the neighbor sampling of the node. In the original algorithm, the input adjacency matrix contains the neighbors of all nodes, and the adjacency samples are obtained by sampling the adjacency matrix during the training process.

### 3.4. Related Parameter Settings

The degree *K*(*V*_*i*_) of the vertex *V*_*i*_ is calculated by the following formula:

(14) $$\begin{array}{c} k\left(v_{i}\right)=\sum_{i=1}^{n}a_{ij}. \end{array}$$

In a hypergraph, the overdegree of vertex *V*_*i*_ is equal to the number of networks with vertices, and represents the number of vertices. Then the overdegree of vertex *V*_*i*_ is expressed as

(15) $$\begin{array}{c} d_{H}\left(v_{i}\right)=\sum_{i=1}^{m}c_{ij}. \end{array}$$

The partitions should satisfy the following balance constraints:

(16) $$\begin{array}{c} W\left(N_{i}\right)\leq \left(1+\varepsilon \right)W_{avg},\;i\in \left(1,k\right). \end{array}$$

The set of vertices in the replicated state within the partition is represented as because the replicated vertices are the communication channels of the partition, so the communication overhead is mainly related to these vertices.

(17) $$\begin{array}{c} C\left(H,\prod \right)=\sum_{v_{i}\in V_{R}}c\left(v_{i}\right),\\ C\left(H,\prod \right)=\sum_{v_{i}\in V_{R}}\left(\lambda \left(v_{i}\right)-1\right)c\left(v_{i}\right). \end{array}$$

After defining the metric *C*(*H*, *π*) of hypergraph partitioning, the optimization problem of partitioning is transformed into finding an optimal partition *π*, which satisfies:

(18) $$\begin{array}{c} \Pi^{*}=\arg\underset{\Pi }{\min}C\left(H,\Pi \right),\\ \text{s.t}.W\left(N_{i}\right)\leq \left(1+\varepsilon \right)W_{ug},\;i\in \left(1,k\right). \end{array}$$

In the network set *N* of a given hypergraph *H*(*V*, *N*), select the smallest number of networks that can contain all vertices:

(19) $$\begin{array}{c} \min,\left(\left|N^{*}\right|\right),N^{*}=\left\{n_{1},n_{2},\ldots ,n_{m}\right\}\subseteq N,\\ s.t.,\;\left\{n_{1}\cup n_{2}\cup \ldots \cup n_{m}\right\}=V. \end{array}$$

In order to avoid falling into the local optimal solution in the process of increasing the network, a random selection is added.

(20) $$\begin{array}{c} w\left(n_{i}\right)=\frac{c\left(n_{i}\right)}{\sum_{n_{i}\in N}c\left(n_{i}\right)}. \end{array}$$

Similarly, in order to avoid falling into a local optimal solution in the process of deleting the network, a random selection process is also needed. The probability of choosing to delete a certain network *n*_*i*_ is

(21) $$\begin{array}{c} w\left(n_{i}\right)=\frac{d\left(n_{i}\right)}{\sum_{n_{i}\in N}d\left(n_{i}\right)}. \end{array}$$

For the hypergraph partition algorithm based on hyperedge partitioning, the cutting metric and balance also play an important role in the evaluation of partition quality, but there are different definitions.

The measurement of hypergraph partition quality reflects the communication cost between partitions. There are two related indicators: one is the vertex cut metric—this metric calculates the number of vertices cut. In particular, vertices with two or more copies are in a cut state. Vertex cutting indirectly affects the communication cost required to segment the hypergraph. The second is the communication cost measurement (measure of the number of copies): this measurement calculates the number of times a vertex must be copied. This is related to the total number of copies of all vertices in the cutting state. At the same time, the number of copies directly affects the communication cost between different partitions of hypergraph. Since the modification of a vertex should be propagated to all its copies to maintain consistency, there are also two metrics for judging the balance of the hypergraph partition: one is the imbalance ratio; the other is the predetermined imbalance in the initialization phase ratio *s* limits the maximum imbalance level of the partition result. The maximum balance constraint of the hypergraph partition is defined by the formula. The balance metric is defined as follows:

(22) $$\begin{array}{c} \theta =\frac{\left(W_{\max}-W_{oug}\right)}{W_{avg},W_{\max}}=\underset{i\leq i\leq k}{\max}\left\{W\left(N_{i}\right)\right\}. \end{array}$$

Then, the standard deviation of the partition size is calculated as follows:

(23) $$\begin{array}{c} \mathrm{NSTDEV}=\sqrt{\frac{{\sum_{i=1}^{k}\left(\left|P_{i}\right|/\left|P\right|/k-1\right)}^{2}}{k}}. \end{array}$$

Normalize the size, such a size partition means that one has

(24) $$\begin{array}{c} \frac{\left|P\right|}{k}=\sum_{n_{j}\in N}\frac{\left|\mathrm{Vectics}\left(n_{j}\right)\right|}{k}. \end{array}$$

### 3.5. Key Technologies of Medical Intelligent System

#### 3.5.1. Data Storage Technology

One of the key technologies of the intelligent medical monitoring service system is data storage technology. The main methods of data storage include: storing data in files, storing data in remote storage space through network transmission, and storing data in databases. File storage read data flow, file storage method is easy to operate but the security of data storage is low, data permissions depend on file permissions, and it is easy to be attacked. Network storage can generally be understood as cloud storage, that is, the use of network transmission to realize data reading and writing, and the amount of data that can be stored is relatively large. However, when data operation is realized through network transmission, network abnormalities and network delay problems will inevitably occur. The operating performance of network storage is poor.

Relational database is a two-dimensional relational storage that converts data into rows and columns. Row storage is to store each row of data continuously, which is equivalent to storing all the attributes of an entity as a unit. The main advantage of row storage is to facilitate assembly. For query results, commonly used row storage databases are MySQL and Oracle. Corresponding to it is the columnar storage method in nonrelational databases, which stores the data in each column continuously, which is equivalent to storing the same attributes in each entity as a unit. The main advantage of columnar storage is that there is no need to add indexes, and each column involved in the query condition can be used as an index during query. Commonly used columnar storage databases are Hbase and Vertica.

Medical data has privacy, and data security is very important. Because the data security of file storage and network storage is not easy to control, the system uses database storage. Since the use of a relational database can realize the control of operational transactions, a relational database is selected. MySQL supports subdatabase and subtable operations. According to subtable routing, data is routed to different tables for storage separately, which will be suitable for data storage in medical systems. The final system adopts MySQL database to realize data storage.

#### 3.5.2. Real-Time Message Transmission Technology

The surgical management function needs to display the real-time patient medical data collected by monitors, ventilators, syringe pumps, and other equipment. It is necessary to realize that each time the gateway transmits the collected monitoring data to the server and the client, both the server and the client can be received in time, the most important thing to realize this function is to realize real-time data transmission.

The key to real-time data transmission is to maintain a long connection between the message sender and the receiver, to avoid the need to establish a connection with the receiver before each message is sent, and to reduce the message sending delay. Commonly used real-time messages are implemented based on the message publish/subscribe model. One party publishes a message, and multiple parties receive messages from the topic in real time by subscribing to the topic. The producer and consumer of the message are not directly coupled together, but relay the message through an intermediate agent. The producer publishes the message to the server, and the server push messages to consumers who subscribe to the corresponding topic. This transmission process is one-to-many. A producer sends a message. As long as the consumer subscribed to the topic can receive the message, there can be multiple consumers.

#### 3.5.3. Real-Time Video Transmission Technology

In the process of surgical monitoring, it is necessary to realize the function of medical staff to remotely view the live video and the screens and data of all medical equipment on the monitoring system workstation to facilitate remote consultation and provide diagnosis and treatment opinions. The key technology to realize this function is real-time video transmission technology.

The general model of general video live broadcast first needs to collect live video streams by means of camera capture, screen recording, and device push streaming. Then the video is encoded by the video encoder. Because the video directly collected by the device is very large, the transmission time is very poor, and the required transmission bandwidth is also large, which cannot be directly transmitted. Therefore, the video compression code must be converted into direct transmission. Currently popular are H.264, AVC, and H.265 video encoders. Then the video encoder pushes the live stream to the streaming media live server. Compared with other live broadcast protocols, the RTMP protocol has high real-time performance, and the delay is generally stable within 3 seconds, which meets the real-time requirements of surgical video live broadcast. When using the RTMP protocol to transmit video, the video is compressed and encoded into FLV format and provided in the form of HTTP. Because it is a long connection based on TCP, there is no need to repeatedly establish a connection each time the video is transmitted, so the delay is relatively low. It is suitable for the low-latency requirements of live video broadcast during surgery.

## 4. The Design and Realization of an Orthopedic Clinical Nursing Medical Intelligent Treatment System

### 4.1. System Requirement Analysis

As shown in Figure 5, the intelligent monitoring system is mainly composed of the hardware part of the intelligent monitoring gateway and the software part of the intelligent monitoring service system. The intelligent monitoring service system includes two parts: the intelligent monitoring system server and the intelligent monitoring system client. The intelligent monitoring gateway realizes the adaptation of monitoring equipment and the collection of medical data, and the intelligent monitoring service system provides service layer resources to realize the effect display of the page.

The intelligent monitoring gateway realizes the adaptation of different medical monitoring equipment and converts different data protocols into a unified data protocol. Push the patient's physiological data collected by the medical monitoring equipment to the upper server and client in real time, so that the medical staff can better understand the patient's vital signs changes during the operation. Push the alarm information collected by the device during the operation to remind the medical staff to pay attention to the abnormal condition of the patient in time. The server of the intelligent monitoring system carries the interactive functions of various data upstream and downstream of the monitoring system gateway side and the intelligent monitoring system client back-end management system, and performs intraoperative patient physiological data collection, management, query, and statistical analysis. Provide real-time message push service, live streaming service, and message queue function. Realize authority control, fine-grained control system user authority.

### 4.2. System Function Module Design

After a detailed demand survey, the functional modules of the system were designed according to the surveyed system requirements. The main functions of the system can be divided into system management module and medical management module. The system management module includes: authority management and monitoring module; and the medical management module includes: equipment management, gateway management, patient management, surgery management, central monitoring function, and alarm management. The functional module diagram of the intelligent medical monitoring service system is shown in Figure 6.

#### 4.2.1. System Management

The authority management module is responsible for realizing the related information management functions of users and authorities in the system. The preliminary investigation found that the medical staffs in the hospital are divided into different types, and each type of medical staff has different authority. Therefore, the system first needs to have a basic authority management module to divide users into different roles, and assign operation functions to each role according to the type of role. To access the system, the login function must first be implemented. Provide users with multiple login methods to facilitate users to quickly log in to the system. In addition, the login page also needs to have a “remember me” function to improve user experience.

#### 4.2.2. Medical Management

The equipment management module is responsible for centralized management of different types of equipment in the hospital. Different types of equipment are distinguished for management. This module includes not only the management of basic information of the equipment itself, but also the management of equipment type information.

The gateway management module is responsible for the unified management of gateways used in various scenarios in the hospital. The medical equipment in each ward sends the collected physiological data to the gateway, and then the gateway sends it to the server. Therefore, the gateway is the key hub for data transmission. This module provides gateway and gateway-type management functions to realize unified management of gateways.

The patient management module is responsible for the management of patient information. In order to realize the digitization of medical information, patient information should be stored persistently, and the operation of patient information is realized in this module.

The operation management module is responsible for the management of basic information and surgical procedures in the operating room. Design the intraoperative monitoring function to monitor and manage the medical process through real-time data online display and video online monitoring methods, and assist medical staff in real-time intraoperative monitoring and guidance of patients.

### 4.3. System Implementation

#### 4.3.1. User Management Function

The user management module mainly implements user-related basic information operation functions and user authority configuration functions. After viewing the user information, other operations can be performed, and the subsequent judgment nodes, respectively, judge to perform the write operation related to the user's basic information, the write operation of the user account status, or the operation of assigning user roles. When all the above processes are executed, the user management process ends.

In the user management page, the user's detailed information can be displayed visually using a table, and the department role can be quickly filtered according to the department through the tree structure of the organization department. The last column of each row displays the operations that can be performed on the current row, including modification and deletion. Intelligent operation of this bank information during operation will not affect other bank information. The buttons for adding users and querying users are displayed separately in the button row above the table because they are not only for single row operations but for full table operations. Personnel changes in hospitals are common. In order to control the timely release of permissions for resigned users, the functions of freezing user accounts and unfreezing user accounts are designed to flexibly control system users. These two function buttons need to be displayed on the page.

#### 4.3.2. Patient Management Function

The patient management module is a basic module of a medical system, responsible for the function of operating basic patient information. After viewing the patient information, you can continue to perform other operations, and the subsequent judgment nodes respectively determine that the write operation of the patient's basic information, the related read operation of quality control management, or the marking operation of the patient are to be performed. After all the above processes are executed, the patient management process ends.

The patient's basic information is displayed in a list on the patient page. You can add basic patient information by clicking the Add button. The operation column at the end of each row can modify or delete the content of this row. In order to view the patient's intraoperative quality control record information and monitoring record information, a monitoring record column and quality control record column need to be added to the list. In each line, a hyperlink button that can jump to the patient's quality control record page and monitoring record page is displayed. Some patients have conditions worthy of special attention and need to design the function of marking patients to achieve special marking of patients. Corresponding to this function is the function of canceling patient marking.

#### 4.3.3. Operation Management Function

*(1) Operating Room Management*. Operation flowchart of the basic functions of the operating room. In this process, viewing the current operating room information is a process that will definitely be performed. You can continue to perform the operation of adding, modifying and deleting the basic information of the operating room. After the execution of the above process, the process of operating room management ends. The operating room page in the system is displayed. In order to facilitate the viewing of the current operating room usage status, if there is a patient currently undergoing surgery, the operating room will be displayed in blue on the page, and the current operating patient, medical record number, and anesthesiologist will be displayed. If there is no patient undergoing surgery in the current operating room, the operating room on the page is displayed in gray.

*(2) Surgical Process Management*. The design of surgical process management is quite complicated, because surgery needs to be performed in accordance with the process, so the functions in the surgical management module also need to be designed strictly in accordance with the surgical process. First, arrange the information of the patients who will be operated on that day in a certain operating room. After the arrangement, the status of these patients will be the waiting state. When it is the turn to perform surgery on a certain patient, the patient state is changed to the state of admission. In order to record the patient's operation time node in the system in detail, the anesthesia start click function is designed, and the system records the anesthesia start time after clicking. After anesthesia, start the operation process for the patient, design the operation start click function, after clicking, the system records the start time of the operation, and at the same time issues real-time monitoring data transmission and real-time monitoring video transmission commands to the gateway to notify the gateway to start transmission. Design the operation end click function, click when the operation is over, the system will record the end time of the operation. Design anesthesia end click function, click when the anesthesia is over, the system will record the anesthesia end time. After the above procedures are executed in sequence, it means that the patient's surgical process is over. If the patient's state is changed to the out-of-room state, the next patient can be scheduled for surgery.

*(3) Central Guardianship Management*. On the basis that the intraoperative monitoring function has been realized, in order to facilitate the medical staff to monitor the operation conditions of multiple operating rooms, a central monitoring function is designed to present the operation scenes of multiple operating rooms on the same screen. First select the operating room to be centrally monitored and the page layout view is several rows and several columns.

After multiple operating room views are displayed on the same screen, in order to facilitate the page to clearly display the intraoperative monitoring status, the intraoperative single split-screen monitoring interface display is changed to display only the basic patient status and the screen video of the monitor by default. Click the display switch button below each view to switch the current monitoring device.

#### 4.3.4. Device and Gateway Management Functions

The design of device management and gateway management is very similar. It realizes the function of persistent operation of related information of the device or gateway. The flowchart of device/gateway type management is similar to that of device/gateway management. Viewing basic information is both. A process will definitely be executed. In the device/gateway management flowchart, two main judgment nodes respectively judge whether to enter the process of viewing detailed information or entering the process of writing basic information. Directly determine the type of write operation in the device/gateway management process. After all the above processes are executed, the process ends.

### 4.4. System Test

#### 4.4.1. System Function Test

Enter different test data according to the function to be tested, and check whether the result of the test function meets expectations. According to the complexity of the function, the amount of input test data is also different. The number of test inputs for simple modules is set to 5, and the number of test inputs for the core modules of the system is set to 10. In order to fully test the quality of the function, the test input data must include both normal data and illegal data that may cause abnormal functions.

During the test, test separately according to the system modules, and first test the function of the authority management module of the system. Since the frequency of use of permission management is not very high, it is mainly used to create new roles, or to redistribute permissions after changing role permissions, so there is no need to consider the concurrency of operations, and only need to test the accuracy of the function. The permission management test process is shown in Table 1. Here, the function test process of adding a role is selected as an example for display.

After the permission management function test is passed, the user management function will be tested. The medical staffs in a hospital are all users of the system, and the order of magnitude is at most thousands or tens of thousands, so there is no need to consider the storage of user data in the database. The operation functions of user management are basically routine operations, and there is no need to consider concurrency issues, just test the feasibility of the function. The user management test process is shown in Table 2.

In the hospital, the operation of patients is more frequent, and there may be two or more medical staff operating the same patient information. During the test, two browsers need to be used to test the relevant functions of patient management at the same time to simulate concurrent scenarios. Test whether the test result is correct.  Table 3 shows the test process of patient management-related functions.

Surgical management is the most important function in the system, including the addition, deletion, modification, and inspection of the operating room, as well as the patient's intraoperative monitoring. Therefore, it is necessary to test whether the operation of the data processing in the operating room is correct, and to test the patient's intraoperative monitoring. Whether the key time node trigger operation in the surgical procedure on the page is correct, and whether the real-time video display and real-time data display are normal. Multiple operations will be performed at the same time in the hospital. In order to simulate the online scene as much as possible during the test, the browsers of two computers are used to test the operation management function. The operation management function test process is shown in Table 4.

Since the function of the gateway management module is similar to the function of the device management module and both are regular data operation functions, the functions of the two modules are tested together, and no concurrent test is required, only the correctness of the operation result is tested. The test process of gateway and device module is shown in Table 5.

The alarm-type management in the alarm management module needs to test whether the addition, deletion, modification, and checking of the alarm type are correct. The alarm information is the real-time alarm information sent by the monitoring device collected by the gateway and sent to the upper layer through the publish/subscribe message mode. The monitoring device needs to simulate the real-time alarm information to test whether the operation details page can receive the real-time alarm information. After receiving the alarm information, test whether the operations of confirming the alarm information, processing the alarm information, and deleting the alarm information are normal. The test process of the alarm management module is shown in Table 6.

The test result is shown in Figure 7. The test pass rate of each module is 100%. The authority management module can realize the distinction of multiple roles in the system and complete the control function of system authority. The user management module can realize the management of basic user information and account status in the system.

### 4.5. Analysis of Orthopedic Clinical Nursing Path

In the context of the current population aging, the incidence of various orthopedic diseases continues to increase. Combining with the past experience in orthopedic nursing management, it can be known that the complexity of orthopedic nursing work is reflected in the higher requirements of orthopedic treatment plans for nursing work. Surgery is a common method of orthopedic treatment. The traumatic stress brought about by this invasive treatment method will further affect the activity function of orthopedic patients. If there is a lack of perfect perioperative care plan, the prognosis of orthopedic patients may be affected to some extent. Most patients need to stay in bed for a long time, and the risk of complications is higher. Due to long-term bed rest, it is easy to cause pressure sores, constipation, infection, and other problems due to long-term local skin pressure, slower gastrointestinal motility, and decreased immune function. This puts forward higher requirements for the prevention and control of related complications in nursing work. Clinical nursing path is a standard process of diagnosis and treatment with scientific and chronological characteristics. This type of nursing method takes the past successful nursing experience as a reference, through a comprehensive summary and analysis, formulates the best nursing plan that meets the needs of the patient, and applies it to nursing practice. In orthopedic nursing, clinical nursing pathway intervention methods require orthopedic nursing staff to jointly formulate orthopedic nursing pathway tables, and in the process of implementing nursing management with reference to the pathway tables, promptly identify and discover the parts of the pathway tables that need improvement, and combine the actual needs of patients. Appropriate adjustments have been made to the content of the path table to ensure the quality of care for orthopedic patients.

## 5. Conclusion

In orthopedic nursing, the application advantages of clinical nursing path are: (1) Relieve pain. On the one hand, fractures can cause more obvious local pain; on the other hand, after surgical treatment, this traumatic treatment method can cause incision pain. Conventional care mostly uses drug analgesia to relieve the pain symptoms of patients, but this analgesic intervention method has a short duration and has limited pain reduction effects. After the introduction of clinical nursing pathways, nursing staff can effectively improve patients' pain conditions through nondrug analgesia and drug analgesia during the critical period of postoperative pain during the second to fourth days after surgery according to the requirements of the pathway table. The results of this study showed that 1 week after nursing, the pain VAS score of the path group was lower than that of the control group. (2) Reduce the risk of complications. Routine care takes as the main goal to ensure the smooth progress of surgical treatment, while the clinical care path takes the causes of complications such as constipation and infection and the period of high incidence as the basis, and formulates good preventive diet care and incision care programs. In this study, the incidence of complications in the pathway group was lower than that in the control group. (3) Promote the recovery of patient's activity function. Combining with previous orthopedic nursing experience, it can be known that the main factors affecting the recovery speed of patients' activity function are patients' cognitive errors and insufficient exercise compliance. The clinical nursing path requires the head nurse to lead the nursing staff to fully analyze the countermeasures of the above-mentioned influencing factors, and finally determine the perioperative nursing plan consisting of preoperative visits and postoperative personalized rehabilitation exercises.

## Figures and Tables

**Figure 1:** The difference between the random sequence generated by BFS red and DFS blue in the random walk sequence.

**Figure 2:** Power law distribution curve of PPI and Reddit data set.

**Figure 3:** The final effect of PPI and Reddit neighbor sampling.

**Figure 4:** The heat map of the number of edges after the division and the distribution of node degree.

**Figure 5:** The composition of the intelligent monitoring system.

**Figure 6:** Functional module diagram of the medical monitoring service system.

**Figure 7:** Histogram of test results.

**Table 1:** Authority management test process.

Test function	Test input	Expected outcome
Add role	Add 3 existing role information in the system; 3 role information with incomplete information; 3 existing role information in the system; directly save once without filling in any information;	The role list shows that there is no role information in the 3 systems just added, the newly added role with incomplete information will give a “Incomplete information” prompt, and the newly added system will prompt “the role already exists,” do not fill in the information to save the prompt required fields

Rights profile	Select an existing role, associate several permission function points for the role, and test 10 times	Users associated with the role can operate the functions corresponding to the permissions configured for the role, but cannot operate the functions corresponding to the unconfigured permissions

Search role	Enter the role name 3 times, enter 2 other search terms	Only the role information that meets the search criteria is displayed in the role information table

Modify selected role	The role information is modified 3 times normally, all fields are blank when one modification is made, and some fields are blank when one modification is made	Normal modification succeeds in modifying the information of the role. When modifying, if the field is left blank, the corresponding required field will be prompted

Delete selected role	Select an existing role, delete the role, test 5 times	The selected role was deleted successfully

**Table 2:** User management test process.

Test function	Test input	Expected outcome
Add user	Add 3 user information already in the system; 3 user information with incomplete information: 3 user information already in the system; directly save once without filling in any information;	The user list shows that there is no user information in the 3 systems just added. The test with incomplete information gives a “Incomplete information” prompt, and the user already exists in the newly added system prompts “the user already exists,” do not fill in the information save prompt required fields

Initialize user password	Select an existing user, reset the user's login password, and test 5 times	The user successfully logged in to the system with the initial password

Disable user	Select a disabled account and test 2 times; test the account in normal state 3 times	Failed to log in to the system with a disabled user account, prompting that the account has been disabled

Unblock user permissions	Select a normal account and test 2 times; test the disabled account 3 times	You can successfully log in to the system with an account that has been lifted

Role assignments	Select an existing user, assign certain roles to the user, test 5 times	The user can operate the permission function points corresponding to several associated roles, but cannot operate other functions without permission

Search for users	Enter the username 3 times and other conditions 2 times	The page will display the information of all registered users that meet the input conditions

Modify selected user information	User information is modified 3 times normally, all fields are blank when one modification is made, and some fields are blank when one modification is made	Normal modification succeeds in modifying the user's information. When modifying, if there are fields left blank, the corresponding required fields will be prompted

Delete selected users	Select the user and delete it, test 5 times	Deleted users are not displayed in the user list

**Table 3:** Patient management test process.

Test function	Test input	Expected outcome
Search for patients	Enter the username 3 times and other conditions 2 times	Patients who meet the search criteria are displayed in the list

Add patient	Add 3 patient information already in the system: 3 patient information with incomplete information: 3 patient information already in the system; directly save once without filling in any information:	The user list shows that there is no user information in the 3 systems just added. The test with incomplete information gives a “Incomplete information” prompt, and the user already exists in the new system prompts “user already exists,” do not fill in the information save prompt required fields

Modify selected patient	The patient information is modified 3 times normally, all fields are blank when one modification is made, and some fields are blank when one modification is made	The patient's information is successfully modified in normal modification, and the corresponding required fields will be prompted when the fields are left blank during modification.

Delete selected patient	Select an existing patient, delete the patient, and test 5 times	Can't find the deleted patient information in the patient information table

View selected patient monitoring records	Check the monitoring record of a patient, test 5 times	View the details of the patient's monitoring record

View quality control records of selected patients	Check the quality control record of a certain patient, test 5 times	View the details of the patient's quality control record sheet

**Table 4:** Hand wood management function test process.

Test function	Test input	Expected outcome
Add operating room	Add 3 tests in the operating room that do not exist in the system, and 2 tests in the existing operating room	Add an operating room that does not exist in the system, and the newly added operating room will be displayed on the page. Add an existing operating room, indicating that the operating room already exists

View selected operating rooms	Set the push streaming address of the video encoding box and the webcam to keep it in the live streaming state, and connect different types of medical equipment to the gateway for data collection. Select an operating room, enter the operating room details page, and test 5 times	You can enter the operating room to view the scene of the operation, trigger operations at key time nodes in the operation process; view monitoring records and quality control records; view the operation scene, anesthesia machine parameters, syringe pump parameters, monitor parameters, etc.

Modify the selected operating room	User information is modified 3 times normally, all fields are blank when one modification is made, and some fields are blank when one modification is made	Normal modification succeeds in modifying the information of the operation room. When modifying, if there are fields left blank, the corresponding required fields will be prompted

Delete the selected operating room	Select an operating room and delete the operating room, test 5 times	The deleted operation room is no longer displayed on the operation management page

**Table 5:** Gateway and equipment module test process.

Test function	Test input	Expected outcome
Basic operation functions of the gateway/device type	Add gateway/device type information in the system, modify the selected gateway/device type information, delete the selected gateway/device type, and query the gateway/device type information in the list. A total of 10 tests	Can realize the basic function processing of the gateway/device type

Basic operating functions of the gateway/device	Add gateway/device information in the system, modify the selected gateway/device information, delete the selected gateway/device, and query the gateway/device information in the list. A total of 10 tests. In the device information table, click the “device discovery” button	Can realize the basic function processing of the gateway/device

Request device discovery	Button, request the server to actively discover the device, request a different medical device each time, test 10	The gateway can receive commands requesting active device discovery

**Table 6:** Test process of alarm management module.

Test function	Test input	Expected outcome
Basic operation function of alarm type	Add alarm type information in the system, modify the selected alarm type information, delete the selected alarm type, and query the alarm type information in the list. A total of 10 tests	Can realize the basic function processing of the alarm type

The gateway sends real-time alarm information	Use monitoring equipment to produce an alarm if the equipment is not connected properly, and the gateway will collect it and send it to the upper layer for 10 tests	The alarm information plus 1 message is received on the operation room details page, and the alarm information of the device just now is displayed in the alarm details page list

Modify the status of unconfirmed alarm information	Modify the status of unconfirmed alarm information to “confirmed” status, test 10 times	The modified alarm has been changed to the confirmed state

Delete alarm information	Delete selected alarm information, test 10 times	The deleted alarms cannot be found in the list

## Data Availability

The data used to support the findings of this study are available from the corresponding author upon request.
